The article "Combination of preoperative fibrinogen and neutrophil to lymphocyte ratio is a predictive prognostic factor in ESCC and AEG systematic review" was published in 2019. Journal: Biosci Rep.

# Combination of preoperative fibrinogen and neutrophil to lymphocyte ratio is a predictive prognostic factor in ESCC and AEG systematic review

**DOI:** 10.1042/BSR20190480

**Published:** 2019-10-15

**Authors:** Guo Tianxing, Pan Xiaojie, Zhu Lihuan, Huang Yangyun

**Affiliations:** Department of Thoracic Surgery, Fujian Provincial Hospital, Provincial Clinical College of Fujian Medical University, Fuzhou City 350001, Fujian Province, China

**Keywords:** esophageal squamous cell carcinoma, fibrinogen, neutrophil to lymphocyte ratio, prognosis

## Abstract

**Objective:** Cancer-associated systemic inflammation response and hyperfibrinogenemia play crucial roles in cancer progression and prognosis. In the present study, we assessed the clinical value of the preoperative fibrinogen and the neutrophil to lymphocyte ratio (NLR) in patients with esophageal squamous cell carcinoma (ESCC) and adenocarcinoma of the esophagogastric junction (AEG).

**Methods:** Three hundred and fifty-six patients who underwent curative surgery were retrospectively analyzed. Univariate and Multivariate Cox analyses were performed to evaluate the prognostic indicators for overall survival (OS). The optimization cut-off values for fibrinogen and the NLR were 3.09 g/l and 1.89, respectively. The fibrinogen and the NLR (F-NLR) index was 2 for patients with high fibrinogen (≥3.09 g/l) and elevated NLR (≥1.89), whereas those with one or neither were indexed as 1 or 0, respectively.

**Results:** The F-NLR score was significantly associated with tumor size (*P*<0.001), and pathological stage (*P*=0.010). The 5-year OS rates in F-NLR groups 0, 1 and 2 were 69.1, 42.6, and 31.9%, respectively (*P*<0.001). Multivariate analysis showed that the tumor size (*P*<0.001), pathological stage (*P*<0.001), and F-NLR (*P*<0.001) were independent prognostic factors for OS. **Conclusions:** The preoperative F-NLR score is an independent prognosis indicator for patients with ESCC and AEG.

## Introduction

Esophageal cancer is one of the common aggressive malignant tumors, with a high ratio of tumor recurrence and mortality [1], esophageal squamous cell carcinoma (ESCC) occupies major portion [2]. Adenocarcinoma of the esophagogastric junction (AEG), is a representative malignancy located between the esophagus and stomach, and was originally characterized by Siewert [3]. It was well-known to have unique clinicopathological features and biological behavior. In recent decades, the incidence rate of AEG gradually rose globally, particularly in the western countries [4]. Although the therapeutic methods have improved, such as surgery, surgery with adjuvant chemotherapy, radiotherapy, or a combination of these treatments, the prognosis of ESCC and AEG patients is poor [5]. Therefore, it is important to search suitable clinical prognostic factors to supply more accurate and precise evaluates of survival, extremely important in high-fatality malignancies. This can both enhance outcomes and decrease costs by better choosing patients for eligible treatment [6].

The article "Combination of preoperative fibrinogen and neutrophil to lymphocyte ratio is a predictive prognostic factor in ESCC and AEG systematic review" was published in 2019. Journal: Biosci Rep.

Cancer-related systemic inflammatory response plays an important role in the progression and outcome of tumors [7,8]. Several common inflammation-based prognostic scoring systems, such as the neutrophil to lymphocyte ratio (NLR) and platelet to lymphocyte ratio (PLR), have been reported to have prognostic value in various cancers, and the high score of NLR and PLR were considered bad prognostic [9,10]. In addition, the hemostatic also plays a key role in cancer progression and metastasis [11,12]. Liver-produced fibrinogen is a key factor in the hemostatic cascade. Recent studies have confirmed that high fibrinogen levels correlate with cancer progression, poor response to chemotherapy and adverse prognostic outcome in various malignancies [13,14]. Recently, several studies analyzed a new scoring system, that is, combining preoperative fibrinogen and the NLR (F-NLR). F-NLR has been demonstrated to be a significant prognostic marker in several types of cancers, such as non-small cell lung cancer and gastric cancer [15,16]. Therefore, the current study aimed to evaluate the prognostic value of F-NLR in patients with ESCC and AEG.

## Materials and methods

### Patients

We performed a retrospective clinical database of 367 patients with ESCC or AEG who underwent curative surgery at Fujian Provincial Hospital, Provincial Clinical College of Fujian Medical University between January 2007 and December 2016. The entire 367 patients were pathologically confirmed to ESCC or AEG, and patients with other tumor types were precluded from this research. Due to majority patients who received neoadjuvant chemotherapy and/or radiotherapy that could have influenced the blood results, 11 patients who had undergone neoadjuvant chemotherapy and/or radiotherapy were excluded. Finally, 356 patients with AEG or ESCC eligible for analysis. Clinicopathological parameters and laboratory inspections of the patients were acquired from the medical records, including sex, age, tumor size, tumor location, histologic differentiation, surgical procedure, TNM stage and blood cell count. The TNM stage was applied according to the 8th TNM classification of American Joint Committee on Cancer (AJCC) staging manual. The work has been reported in line with AMSTAR (Assessing the Methodological Quality of Systematic Reviews) Guidelines.

The article "Combination of preoperative fibrinogen and neutrophil to lymphocyte ratio is a predictive prognostic factor in ESCC and AEG systematic review" was published in 2019. Journal: Biosci Rep.

### F-NLR evaluation

Hematological laboratory measurements including neutrophil count, lymphocyte count, and fibrinogen concentrations, were extracted from the daily blood test administered in the week before surgery. The NLR was defined as dividing the neutrophil count by the lymphocyte count. According to the Youden index by Receiver operating characteristic (ROC) curve, the most appropriate cut-off threshold was found as 3.09 g/l for plasma fibrinogen and 1.89 for NLR; for these values, an area under the curve (AUC) as 0.628 and 0.585, respectively. Based on these cut-off values, the F-NLR score was classified as follows: F-NLR score of 2 [both a hyperfibrinogenemia (≥3.09 g/dl) and high NLR (≥1.89)], 1 [either hyperfibrinogenemia (≥3.09 g/l) or high NLR (≥1.89)], 0 [neither hyperfibrinogenemia nor high NLR].

### Statistical analysis

Statistical analysis was done using SPSS software version 22 (IBM, Armonk, New York, U.S.A.). A two-tailed chi-squared test and Spearman-rho test was used to evaluate differences in categorical variables. Differences between the overall survival (OS) generated by the Kaplan–Meier curves were decided using the log-rank test. OS was defined as the time in months between the date of surgery and the date of death or last follow-up. Univariate and multivariate analyses were carried out by Cox regression models to clarify the independent prognostic factors. All *P*-values were quoted two-sided, and a *P*-value of <0.05 was considered to represent statistical significance.

The work has been reported in line with PRISMA (Preferred Reporting Items for Systematic Reviews and Meta-Analyses) Guidelines.

## Results

### Patient characteristics

A total of 356 patients who were pathologically diagnosed as ESCC or AEG were included in this retrospective analysis (Table 1). All patients underwent curative surgery resection. The present study included 280 (78.7%) male and 76 (21.3%) female, the median age was 62 (range 32–76) years. Patients were categorized into three independent groups as follows: F-NLR = 0, 95 (26.7%) patients; F-NLR = 1, 145 (40.7%) patients; and F-NLR = 2, 116 (32.6%) patients. All 49, 114, and 193 patients presented with pathological TNM stages I, II, and III, respectively. According to tumor location, 129 and 227 patients were classified as having AEG and ESCC, respectively. The median follow-up duration was 48.4 months.

**Table 1:** Characteristics of the recruited patients

Characteristics	Median (25th–75th percentile) or number (%)
Gender	
Male	76 (21.3)
Female	280 (78.7)
Age (years)	
<60	145 (40.7)
≥60	211 (59.3)
TNM stage	
I–II	138 (43.4)
III–IV	180 (56.6)
5-year survival	
Yes	134 (42.1)
No	184 (57.9)
Tumor size (cm)	
<5	162 (45.5)
≥5	194 (54.5)
NLR	2.87 (1.93–5.89)
PLR	164.92 (114.17–241.15)
Fibrinogen (g/dl)	3.32 (0.66–8.06)
Neutrophil	4.21 (3.08–6.28)
Platelet	1.40 (0.93–1.76)
Lymphocyte	222.15 (175.9–273.3)
Albumin (g/l)	43 (39.55–45.58)
Hemoglobin (g/l)	121 (102–133)
	

The article "Combination of preoperative fibrinogen and neutrophil to lymphocyte ratio is a predictive prognostic factor in ESCC and AEG systematic review" was published in 2019. Journal: Biosci Rep.

### Prognostic analysis based on plasma fibrinogen or NLR

Patients with hyperfibrinogenemia had a much worse 5-year OS than those with low fibrinogen (31.4 *vs.* 63.3%, *P*<0.001; Figure 1). Patients with increased NLR had a poorer 5-year OS than those with low NLR (40.4 *vs*. 50.3%, *P*=0.003; Figure 2).

**Figure 1:** Kaplan–Meier survival curves for patients in high fibrinogen and low fibrinogen groups

**Figure 2:** Kaplan–Meier survival curves for patients in high NLR and low NLR groups

### Correlation between F-NLR and clinicopathological factors

The association between the F-NLR score and clinicopathologic features of patients with AEG and UGC is shown in Table 2. There was significant correlation of F-NLR with tumor size (*P*<0.001) and pathological stage (*P*=0.010).

**Table 2:** Univariate and Multivariate analyses of factors for prediction of OS

		Univariate analysis		Multivariate analysis	
	*Wald value*	*P*-value	*Wald* value	*HR value (95% CI)*	*P-*value
Gender (male/female)	1.189	0.276			
Age (<60 years/≥60 years)	1.662	0.197			
NLR	6.521	0.000*	0.008	0.985 (0.699, 1.388)	0.930
Tumor location (ESCC/AEG)	0.860	0.354			
TNM stage (I, II / III)	109.07	0.000*	49.835	2.373 (1.867, 3.017)	0.000*
Differentiation grade (well/moderate/poor)	0.369	0.544			
Albumin (<42 g/l/≥42 g/l)	0.124	0.725			
Tumor size (<5 cm/≥5 cm)	20.56	0.000*	6.480	0.724 (0.564, 0.928)	0.011*
PLR	19.43	0.000	1.684	1.396 (0.843, 2.311)	0.194
F-NLR	44.26	0.000	7.657	1.730 (1.173, 2.551)	0.006*
Fibrinogen (g/dl)	4.965	0.026	0.125	1.083 (0.696, 1.684)	0.724
Hemoglobin (<120 g/l/≥120 g/l)	2.784	0.095			

* was considered to be statistically significant.

### Survival analysis of F-NLR

We conducted the Kaplan–Meier analysis and log-rank test to determine the survival differences between the three groups categorized by F-NLR score. For all the patients, the 5-year OS rates were 69.1, 42.6, and 31.9% for F-NLR = 0, F-NLR = 1, and F-NLR = 2, respectively (*P*=0.001, Figure 3).

**Figure 3:** Kaplan–Meier survival curves for F-NLR score 0 group, F-NLR score 1 group, F-NLR score 2 group

### F-NLR as prognostic factor

To identify the independent prognostic indexes for OS, we carried out univariate and multivariate analyses with a Cox proportional hazard model. In a univariate survival analysis, The tumor size (*P*<0.001), surgical procedure (*P*=0.043), pathological stage (*P*<0.001), and F-NLR (*P*<0.001) were associated with OS. Multivariate analysis demonstrated that the tumor size (*P*<0.001), pathological stage (*P*<0.001), and F-NLR (*P*<0.001) were considered independent prognostic factors for OS (Table 3).

The article "Combination of preoperative fibrinogen and neutrophil to lymphocyte ratio is a predictive prognostic factor in ESCC and AEG systematic review" was published in 2019. Journal: Biosci Rep.

**Table 3:** Relationship between F-NLR and clinicopathologic characteristics

Characteristics	F-NLR			*P*-value
	0	1	2	
Gender				0.581
Female	22	33	21	
Male	73	112	95	
Age (years)				0.056
<60	48	57	40	
≥60	47	88	76	
Tumor size				<0.001
<5 cm	58	65	39	
≥5 cm	37	80	77	
TNM stage				0.010
I-II	55	54	44	
III-IV	40	81	72	
Differentiation grade				0.107
High	30	36	22	
Moderate-Low	65	109	94	
Tumor location				0.158
ESCC	53	98	76	
AEG	42	47	40	

## Discussion

Although surgical techniques and adjuvant treatments has improved, the median survival of ESCC and AEG malignancies remains unsatisfactory [17]. Early diagnosis and treatment are key to increase the OS time of patients. Recent studies revealed that the development of cancer is related to chronic inflammation and hemostatic system [18–20]. In our current retrospective study, we investigated the prognostic value of F-NLR score and the relationship between F-NLR and clinicopathological features in the patients with AEG and EDCC.

Inflammation and immune cells are essential components of the tumor microenvironments. The systemic inflammatory responses play important role in tumor growth, progression, and metastasis by creating a favorable microenvironment and inhibiting anti-tumor immunity [21,22]. The systemic inflammatory responses disrupt the balance of circulating white blood cell components [23]. Thus, it affects the numbers of neutrophils and lymphocytes in leukocyte during cancer progression. The NLR has been recognized as a representative prognostic indicator in various malignancies [24–26].

In addition, more and more studies have demonstrated the association between hemostatic system and cancer progression in recent years. Increasing evidence have suggested that the activation of the hemostatic cascade plays a crucial pathophysiological role in tumor aggressiveness [27]. Fibrinogen is a main acute-phase protein and as an important component of the hemostatic system has been shown to be a necessary regulator of the systemic inflammatory state and malignancy progression [28]. It may mediate the original adhesion of white blood cells to endothelial cells and the release of pro-inflammatory cytokines, thus induce cancer cell proliferation and progression [29]. Hyperfibrinogenemia has been confirmed to be a significant prognostic predictor with tumor progression and poor response to chemotherapy in various malignancies [30].

Therefore, the combination serum fibrinogen and NLR (F-NLR) provides a good prognostic marker for cancer patients. Fibrinogen alone or NLR may have a limited effect on tumor progression. F-NLR increases the adverse effects of F-NLR, ultimately increases the predictive significance of cancer patients. In the current study, we demonstrated that univariate and multivariate analyses revealed that preoperative F-NLR was significantly associated with OS, as well as tumor size and pathological stage, which was consistent with previous study. Based on the Kaplan–Meier method, our study divided the patients into three different risk groups according to the preoperative F-NLR level, and F-NLR score 0 group had a longer survival time. The results suggested that F-NLR might be a reliable prognostic marker. The fact that F-NLR score can be obtained from the routine blood sample makes it practical and inexpensive. Thus, F-NLR may be suitable as a more universally hematological marker than other tumor markers.

The article "Combination of preoperative fibrinogen and neutrophil to lymphocyte ratio is a predictive prognostic factor in ESCC and AEG systematic review" was published in 2019. Journal: Biosci Rep.

The present study had several shortages. First of all, the present study was a single institute, retrospective analysis with a small number of patients. Second, although we restricted some possible mixed factors, the hematologic cell counts can be influenced by several factors. Finally, we were short of the follow-up information for disease-free survival, and our conclusions may be reinforced by using other methods of survival. In the future, we will further improve our study to supply more accurate and precise evaluates of survival.

## Conclusion

The preoperative F-NLR score is an independent predictor of survival in patients who underwent curative surgery for AEG and ESCC. As it is objectively measured and daily available, which may be a useful clinical biomarker for identifying patients at high prognostic risk and planning individualized treatment strategies for patients with AEG and ESCC.

## Availability of data and materials

The datasets used and/or analyzed during the current study are available from the corresponding author on reasonable request.

## Abbreviations

AEG: adenocarcinoma of the esophagogastric junction
ESCC: esophageal squamous cell carcinoma
F-NLR: fibrinogen and the neutrophil to lymphocyte ratio
NLR: neutrophil to lymphocyte ratio
OS: overall survival
PLR: platelet to lymphocyte ratio
TNM: Tumor Node Metastasis
